The article "Overexpression of lncRNA TCTN2 protects neurons from apoptosis by enhancing cell autophagy in spinal cord injury" was published in 2019. Journal: FEBS Open Bio.

# Overexpression of lncRNA TCTN2 protects neurons from apoptosis by enhancing cell autophagy in spinal cord injury

**DOI:** 10.1002/2211-5463.12651

**Published:** 2019-06-04

**Authors:** Xiao‐dong Ren, Chun‐xiao Wan, Ya‐li Niu

**Affiliations:** ^1^ Department of Rehabilitation The General Hospital Tianjin Medical University China

**Keywords:** autophagy, Beclin‐1, miR‐216b, neuronal apoptosis, spinal cord injury, TCTN2

## Abstract

Neuronal apoptosis is the main pathological feature of spinal cord injury (SCI), while autophagy contributes to ameliorating neuronal damage via inhibition of apoptosis. Here, we investigated the role of tectonic family member 2 (TCTN2) long non‐coding RNA on apoptosis and autophagy in SCI. TCTN2 was down‐regulated in the spinal cord tissues of a rat model of SCI and in oxygen–glucose deprivation‐induced hypoxic SY‐SH‐5Y cells, while microRNA‐216b (miR‐216b) was up‐regulated. Overexpression of TCTN2 reduced neuron apoptosis by inducing autophagy, and TCTN2 was observed to negatively regulate miR‐216b. Furthermore, TCTN2 promoted autophagy to repress apoptosis through the miR‐216b–Beclin‐1 pathway, and overexpression of TCTN2 improved neurological function in the SCI rat model. In summary, our data suggest that TCTN2 enhances autophagy by targeting the miR‐216b–Beclin‐1 pathway, thereby ameliorating neuronal apoptosis and relieving spinal cord injury.

**Abbreviations**
3‐MA: 3‐methyladenine
AGO2: Argonaute2
BBB scoring: Basso, Beattie, and Bresnahan scoring
ECL: electrochemical luminescence
lncRNA: long non‐coding RNA
miR‐216b: microRNA‐216b
OGD: oxygen–glucose deprivation
qRT‐PCR: quantitative real‐time PCR
RIP: RNA immunoprecipitation
SCI: spinal cord injury
TCTN2: tectonic family member 2

Apoptosis, also called programmed cell death, refers to an intrinsic pathway of cell death caused by various physiological or pathological signals, and inappropriate apoptosis is closely associated with human disorders 1, 2. Neuronal apoptosis is a main factor of neuronal loss in diverse neurological diseases, especially in neurodegenerative diseases 3. Neuronal apoptosis is one of the primary features observed in spinal cord injury (SCI), leading to a certain degree of neurological damage, necrosis, or autonomic nervous dysfunction 4, 5. However, apoptosis does not function alone in determining the fate of a cell 6. Autophagy, a dynamic process that triggers the self‐digestion of damaged organelles and misfolded proteins in cells, is believed to engage in a complex interplay with apoptosis 7.

In SCI model rats, autophagy has been verified to decrease neuronal damage and promote locomotor recovery, through suppressing neuronal apoptosis after SCI 8. Beclin‐1 protein has been proven to be associated with both autophagy and apoptosis 9. In spinal cord neurons, overexpression of Beclin‐1 remarkably enhances autophagy and reverses mechanical injury‐induced cell apoptosis, suggesting a role of Beclin‐1 in promoting autophagy and protecting neurons from apoptosis in SCI 10. In addition, up‐regulation of Beclin‐1 by vascular endothelial growth factor 165 contributes to increasing autophagy to attenuate SCI 11. These findings identify an essential role of Beclin‐1 in affecting autophagy, neuronal apoptosis, and the subsequent SCI development. Furthermore, Beclin‐1 has been identified as a target of microRNA‐216b (miR‐216b) and the miR‐216b–Beclin‐1 axis regulates both autophagy and apoptosis in human Tenon's capsule fibroblasts 12. The interaction between miR‐216b and Beclin‐1 and its effect on autophagy and apoptosis have not been investigated in SCI.

The article "Overexpression of lncRNA TCTN2 protects neurons from apoptosis by enhancing cell autophagy in spinal cord injury" was published in 2019. Journal: FEBS Open Bio.

Tectonic family member 2 (TCTN2) belongs to the Tectonic (TCTN) family, and mutations in TCTN2 have been recently reported to disturb neural tube development in human and mouse, and loss of TCTN3 causes neuronal apoptosis 13. TCTN2 knockout shows neural tube defects in mouse 14, indicating a crucial influence of TCTN2 on neuronal apoptosis. The binding sites between miR‐216b and the long non‐coding RNA (lncRNA) TCTN2 (transcript: ENSMUST00000100706) predicted with the bioinformatics method imply a potential interaction between them. LncRNAs refer to RNA transcripts with more than 200 nucleotides that do not encode proteins, and they widely regulate gene expression in diverse biological and pathological processes. Based on the above findings, we infer that TCTN2 may participate in the neuronal apoptosis via interplay with miR‐216b to affect its target, Beclin‐1. Therefore, we undertook this study to explore whether lncRNA TCTN2 plays a role in autophagy and neuronal apoptosis, aiming to illuminate the function of this long non‐coding transcript in SCI progression for the first time.

## Materials and methods

### Animal treatment

All the animal experiments were conducted in accordance with the Guide for the Care and Use of Laboratory Animals of the Chinese National Institutes of Health and approved by the Animal Care Committee of the Genernal Hospital, Tianjin Medical University. Sprague–Dawley rats (200–250 g) were used in the study and to ensure the animals did not suffer unnecessarily at any stage, they were housed in a clean environment with controlled temperature (23–25 °C) and provided with *ad libitum* food and water. SCI models (SCI group, *n* = 6) were constructed according to a previous protocol 15. To relieve pain, rats were anesthetized by intraperitoneal injection with 10% chloral hydrate (3 mL·kg^−1^), and then kept in prone position on the console. A laminectomy at the T9–T10 spinous process was conducted to thoroughly expose the spinal cord. Then spinal cord crush was performed with a 10 g weight dropped from a height of 5 cm to strike the spinal cord surface. The muscle and skin were sutured in layers. Paralysis of the lower limbs, tail swing, and spinal cord hematoma formation were observed in a successful SCI model. Only laminectomy was conducted in sham rats (sham, *n* = 6). After the SCI surgery, the bladder of the rats was massaged twice per day until the spontaneous voiding function of the bowel recovered.

The article "Overexpression of lncRNA TCTN2 protects neurons from apoptosis by enhancing cell autophagy in spinal cord injury" was published in 2019. Journal: FEBS Open Bio.

### Basso, Beattie, and Bresnahan scoring

The motor function recovery of rat was estimated using Basso, Beattie, and Bresnahan (BBB) scoring with a 21‐point open field locomotor scale 8, in which a score of 0 indicates complete immobility and 21 indicates normal motor function. Double‐blinded observation of the rats’ locomotion was carried out respectively at 1, 6, 12, 24, and 48 h after SCI. The hind limb movements, stepping, stability, trunk position, coordination, paw placement, toe clearance, and tail position of the rats were observed and recorded. Two observers blinded to the groups obtained the BBB scores individually for mean value calculation.

### Quantitative real‐time PCR

At 48 h post‐SCI, rats were sacrificed and the spinal cord tissues located 1 cm above and below the injury site were taken for total RNA extraction using Trizol reagent (Thermo Fisher Scientific, Waltham, MA, USA). RNA was quantified with a Nanodrop 2000 system and reverse‐transcribed with a Taqman Reverse Transcription Kit (Thermo Fisher Scientific). Subsequently, SYBR Green Master Mix (Applied Biosystems) was utilized for the quantitative RT‐PCR on an ABI PRISM 7500 sequence detection system (Thermo Fisher Scientific). Oligonucleotide primers were synthesized by Sangon Biotech (Shanghai, China). The relative expressions of TCTN2 and miR‐216b were calculated with the 2^−∆∆*C*t^ method.

### Western blot analysis

Spinal cord tissues were lysed in RIPA lysis buffer (Beyotime, China) containing protease inhibitors. After centrifugation, the supernatant was collected and the protein extraction was separated with 12% SDS/PAGE. Protein was transferred to polyvinylidene difluoride membranes (Bio‐Rad Laboratories, Hercules, CA, USA) and then blocked in Tris‐buffered saline with 5% non‐fat milk for 2 h at room temperature. The membranes were probed with specific primary antibodies (Abcam, Cambridge, UK) against Beclin‐1 and β‐actin at 4 °C overnight. The membrane was washed and incubated in horseradish peroxidase‐bound secondary antibodies for 2 h at room temperature and imaged on a Tanon Chemiluminescence Imaging system with an ECL regent (Thermo Fisher Scientific).

The article "Overexpression of lncRNA TCTN2 protects neurons from apoptosis by enhancing cell autophagy in spinal cord injury" was published in 2019. Journal: FEBS Open Bio.

### Cell culture and hypoxia treatment

The human hippocampal neuron‐derived cell line SY‐SH‐5Y was cultured in Ham's F12 medium supplemented with Eagle's minimum essential medium (EMEM) (1 : 1), 1% non‐essential amino acids, 2 mm glutamine, 15% fetal bovine serum and maintained at 37 °C with 5% CO_2_. An oxygen–glucose deprivation (OGD) assay was performed to mimic the pathological conditions of ischemia for neuronal injury induction through a reduction in the supplement of oxygen and glucose 16. Neurons were incubated in OGD solution in a controlled hypoxic incubator (Thermo Forma, San Jose, CA, USA) with an environment of 94% N_2_/5%CO_2_/1% O_2_ at 37 °C for 1 h. The neurons were then cultured in OGD solution with 5.5 mm glucose at 37 °C with 5% CO_2_ for 24 h for reoxygenation.

### Flow cytometry

After OGD treatment, SY‐SH‐5Y cell apoptosis was measured with an annexin V–FITC/propidium iodide cell apoptosis detection kit (Sigma‐Aldrich, St Louis, MO, USA) followed by flow cytometric analysis. SY‐SH‐5Y cells (2 × 10^5^/well) were seeded in six‐well plates and grown to 70–80% confluence. The cells were harvested and stained with 200 μL annexin V‐FITC and 10 μL propidium iodide, followed by flow cytometric analysis on a flow cytometer (FACSCalibur, BD Biosciences, Franklin Lakes, NJ, USA).

### Cell transfection

The pcDNA‐TCTN2 vector (with pcDNA acting as negative control), miR‐216b mimic and its negative control, pre‐NC, were synthesized by GenePharma (Shanghai, China). These plasmids were transfected into SY‐SH‐5Y cells using Lipofectamine 2000 (Invitrogen) according to the manufacture's manual; 48 h following cell transfection, the expression level of TCTN2, miR‐216b, and Beclin‐1 protein was analyzed.

### RNA immunoprecipitation

Binding between TCTN2 and miR‐216b was estimated with RNA immunoprecipitation (RIP) assay using the RNA‐Binding Protein Immunoprecipitation Kit (Millipore, Boston, MA, USA). SY‐SH‐5Y cells were lysed and the lysate was incubated with Argonaute2 (AGO2) antibody or negative control (normal mouse IgG, Abcam). RNA–protein complexes were immunoprecipitated with protein A agarose magnetic beads and the unbound material was washed off. RNA was extracted by using Trizol reagent (Invitrogen) and quantitative real‐time PCR (qRT‐PCR) was performed to detect the expression of TCTN2. Immunoprecipitation–western blotting was conducted to measure the AGO2 protein level.

### RNA pull‐down assay

RNA pull‐down assay was performed using a Magnetic RNA‐Protein Pull‐Down Kit (Thermo Fisher Scientific). A DNA probe complementary to TCTN2 was synthesized and biotinylated (GenePharma), and 3 μg of streptavidin‐labeled TCTN2 was mixed with protein in Protein‐RNA Binding Buffer. The biotinylated RNA was incubated with cell lysate and magnetic beads. After the beads were washed three times, the RNA‐binding protein complexes were finally eluted and the enriched RNA was determined by qRT‐PCR analysis.

The article "Overexpression of lncRNA TCTN2 protects neurons from apoptosis by enhancing cell autophagy in spinal cord injury" was published in 2019. Journal: FEBS Open Bio.

### Overexpression of TCTN2 in SCI model rat

To verify the role of TCTN2 in SCI progression *in vivo*, an SCI rat model was established. The vector highly expressing TCTN2 named pcDNA‐TCTN2 (volume of 5 μL) and its negative control pcDNA (volume of 5 μL) were injected into the spinal cord of rats (*n* = 6 in each group) using a glass micro‐pipette attached to a pico spritzer (Parker Instrumentation, Fairfield, NJ, USA) 17. BBB scoring was carried out at 1, 6, 12, 24, and 48 h following surgery. Rats were sacrificed at 48 h following SCI and the spinal cord tissues were obtained for the experiments that followed.

### Statistical analysis

spss statistics 21.0 software (IBM Corp., Armonk, NY, USA) was used for statistical analyses. All experiments were repeated at least three times, and all the data are presented as mean ± standard deviation (SD). Two‐group comparisons were analyzed with Student's *t* test, and a value of *P* < 0.05 was considered significantly different.

## Results

### Down‐regulation of TCTN2 in SCI rat model

To evaluate the expression level of TCTN2 in SCI, an SCI rat model was constructed. The neurological function of the SCI rat model was assessed with BBB scoring at 1, 6, 12, 24, and 48 h after SCI. Compared with the rat in sham group (*n* = 6), the BBB score in SCI rat (SCI, *n* = 6) was clearly lower (Fig. 1A). Forty‐eight hours after SCI, the spinal tissue of the rats was isolated and the expression of TCTN2, miR‐216b, and Beclin‐1 protein in the tissue was determined. The expression of TCTN2 was dramatically diminished in spinal tissue of the SCI group (SCI, *n* = 6) when compared with the sham group (*n* = 6), while miR‐216b level was markedly elevated in the SCI group (Fig. 1B). However, the Beclin‐1 protein level was significantly decreased in spinal tissue of the SCI group (SCI, *n* = 6) (Fig. 1C). The results indicated the abnormal expression of TCTN2, miR‐216b, and Beclin‐1 protein in SCI, implying their potential influence on SCI initiation and development.

**Figure 1:** Down‐regulation of TCTN2 in SCI rat model and OGD‐induced neurons and its influence on neuronal apoptosis. SCI rat model (SCI, *n* = 6) was constructed, and the rats in sham group (*n* = 6) served as control. (A) Neurological function of rats was assessed with BBB scoring at 1, 6, 12, 24, and 48 h after SCI establishment. (B) Forty‐eight hours following SCI, the spinal tissue of mice was taken and the expression of TCTN2 and miR‐216b in spinal tissue was quantified with qRT‐PCR. (C) The protein expression of Beclin‐1 was determined with western blot 48 h after SCI. *P < 0.05 compared with the sham group. The error bars indicated SD. The experiments were repeated three times. Comparisons between the two groups were analyzed with Student's *t* test.

The article "Overexpression of lncRNA TCTN2 protects neurons from apoptosis by enhancing cell autophagy in spinal cord injury" was published in 2019. Journal: FEBS Open Bio.

### Down‐regulation of TCTN2 in OGD‐induced neurons and its influence on neuronal apoptosis

SY‐SH‐5Y was treated with OGD to imitate a hypoxic environment, and the expression of TCTN2, miR‐216b, and Beclin‐1 protein in control and OGD‐treated cells was detected. Figure 2A shows that TCTN2 expression was suppressed in SY‐SH‐5Y cells treated with OGD, while the expression of miR‐216b was enhanced. Nevertheless, the protein expression of Beclin‐1 was inhibited in SY‐SH‐5Y cells treated with OGD (Fig. 2B). To assess the influence of TCTN2 on autophagy and neuronal apoptosis, SY‐SH‐5Y cells were divided into five groups: control, OGD, OGD+pcDNA, OGD+pcDNA‐TCTN2, and OGD+pcDNA‐TCTN2+3‐methyladenine (3‐MA), with 3‐MA serving as an autophagy inhibitor. The results indicated that transfection of pcDNA‐TCTN2 recovered the TCTN2 expression that was repressed by OGD, but no difference was noted after 3‐MA treatment (Fig. 2C). An evaluation of apoptotic status showed that OGD treatment induced apoptosis, pcDNA‐TCTN2 relieved apoptosis caused by OGD, but it was further reversed by 3‐MA treatment (Fig. 2D). Beclin‐1 and LC3II protein expression was restrained with OGD treatment but augmented by TCTN2 overexpression, and then inhibited after 3‐MA treatment (Fig. 2E). The protein expression of P62 was increased by OGD but decreased with pcDNA‐TCTN2 transfection, which was finally reversed by 3‐MA treatment; but the LC3I level remained unchanged (Fig. 2E). LC3 is the autophagy‐associated protein that is post‐translationally cleaved and localizes in the cytosol (LC3I) or in autophagosomal membranes (LC3II). Hence detection of LC3II was used to evaluate the abundance of autophagosomes. The above results revealed that overexpression of TCTN2 reduced neuronal apoptosis by inducing autophagy.

**Figure 2:** Cells of the human hippocampal neuron‐derived cell line, SY‐SH‐5Y were grouped into control and OGD for detection of TCTN2, miR‐216b, and Beclin‐1 protein expression. (A) After OGD treatment, the expression of TCTN2 and miR‐216b in SY‐SH‐5Y cells was examined by qRT‐PCR. (B) The protein level of Beclin‐1 was analyzed with western blot. (C) The expression of TCTN2 in SY‐SH‐5Y cells was estimated with qRT‐PCR. (D) SY‐SH‐5Y cell apoptosis was analyzed by flow cytometry. (E) The expression of Beclin‐1, P62, LC3I, and LC3II protein in SY‐SH‐5Y cells was assessed with western blot. *P < 0.05 compared with control; ^#^ *P* < 0.05 compared with OGD+pcDNA; ^&^ *P* < 0.05 compared with OGD+pcDNA‐TCTN2. The error bars indicate SD. The experiments were repeated three times. Comparisons between the two groups were analyzed with Student's *t* test.

The article "Overexpression of lncRNA TCTN2 protects neurons from apoptosis by enhancing cell autophagy in spinal cord injury" was published in 2019. Journal: FEBS Open Bio.

### Interaction between TCTN2 and miR‐216b

The putative binding site between TCTN2 and miR‐216b is shown in Fig. 3A. Their binding and interaction in SY‐SH‐5Y cells were assessed. AGO2 antibody was used in the RIP assay. Compared with IgG, a mass of TCTN2 and miR‐216b was detected with the AGO2 antibody (Fig. 3B). In the RNA pull‐down assay, AGO2 in the pull‐down complex of TCTN2 was analyzed, and miR‐216b was deposited extensively in the pull‐down complex of TCTN2, while a slight increase was observed in the negative control (NC) group (Fig. 3C). These data identified miR‐216b as a target of TCTN2 in SY‐SH‐5Y cells.

**Figure 3:** Relationship between TCTN2 and miR‐216b. RNA immunoprecipitation (RIP) and RNA pull‐down assay were performed to explore the interaction between TCTN2 and miR‐216b in SY‐SH‐5Y cells. (A) Bioinformatics analysis (DIANA) predicted the binding sites between TCTN2 and miR‐216b. (B) RIP assay was performed to determine the binding condition between TCTN2 and miR‐216b, and immunoprecipitation–western blotting was performed to determine whether TCTN2 and miR‐216b are present in the AGO2 protein complex. (C) RNA pull‐down assay was conducted to examine the interaction between TCTN2 and miR‐216b. *P < 0.05 compared with Input or negative control (NC). The error bars indicate SD. The experiments were repeated three times. Comparisons between the two groups were analyzed with Student's *t* test.

### TCTN2 regulates autophagy and apoptosis through the miR‐216b–Beclin‐1 pathway

To investigate the role of TCTN2 and miR‐216b and their interaction in neuronal apoptosis, SY‐SH‐5Y cells were assigned to six groups: control, OGD, OGD+pcDNA, OGD+pcDNA‐TCTN2, OGD+pcDNA‐TCTN2+pre‐NC (the negative control of miR‐216 mimic), and OGD+pcDNA‐TCTN2+miR‐216b mimic. Compared with the control group, miR‐216b expression was promoted by OGD treatment but then inhibited with pcDNA‐TCTN2 transfection, which was further inverted by miR‐216b mimic, while the Beclin‐1 protein expression change was the contrary of that of miR‐216b (Fig. 4A). The protein level of P62 was increased by OGD but decreased with pcDNA‐TCTN2 transfection, which was finally reversed by up‐regulation of miR‐216b. The expression of LC3II protein was decreased with OGD treatment but increased after pcDNA‐TCTN2 transfection, which was finally reversed with overexpressed miR‐216b mimic (Fig. 4B). Neuronal apoptosis induced by OGD was mitigated by pcDNA‐TCTN2 transfection but then inverted by miR‐216b mimic (Fig. 4C). Herein, we showed that TCTN2 regulated autophagy and apoptosis through miR‐216b.

The article "Overexpression of lncRNA TCTN2 protects neurons from apoptosis by enhancing cell autophagy in spinal cord injury" was published in 2019. Journal: FEBS Open Bio.

**Figure 4:** TCTN2 regulated autophagy and apoptosis through miR‐216b–Beclin‐1 pathway. SY‐SH‐5Y cells were assigned to six groups: control, OGD, OGD+pcDNA, OGD+pcDNA‐TCTN2, OGD+pcDNA‐TCTN2+pre‐NC, and OGD+pcDNA‐TCTN2+miR‐216b mimic. (A) Forty‐eight hours after cell transfection, the expression of miR‐216b and Beclin‐1 protein was evaluated with qRT‐PCR and western blot, separately. (B) The expression of P62, LC3I, and LC3II protein in SY‐SH‐5Y cells was assessed with western blot. (C) SY‐SH‐5Y cell apoptosis was estimated with flow cytometric analysis. *P < 0.05 compared with control; ^#^ *P* < 0.05 compared with OGD+pcDNA; ^&^ *P* < 0.05 compared with OGD+pcDNA‐TCTN2+pre‐NC. The error bars indicate SD. The experiments were repeated three times. Comparisons between the two groups were analyzed with Student's *t* test.

### Overexpression of TCTN2 improved neurological function in SCI rat model

To validate the influence of TCTN2 expression on SCI progression *in vivo*, the SCI rat model was intrathecally injected with pcDNA (*n* = 6) or pcDNA‐TCTN2 (*n* = 6) vector. BBB scoring was performed to estimate the neurological function at 1, 6, 12, 24, and 48 h after SCI. Compared with the pcDNA (*n* = 6) group, the BBB score of rats with pcDNA‐TCTN2 (*n* = 6) was clearly elevated from 12 h to 48 h (Fig. 5A). Notably, the expression of TCTN2 was also increased with pcDNA‐TCTN2 introduction, while the miR‐216b expression was reduced (Fig. 5B). P62 protein level was decreased in the pcDNA‐TCTN2 group, while the expression of LC3II protein was clearly elevated (Fig. 5C), implying that autophagy was facilitated by overexpression of TCTN2. These findings demonstrated that overexpression of TCTN2 improved neurological function in the SCI rat model.

**Figure 5:** Overexpression of TCTN2 improved neurological function in SCI rat model. SCI rat model was intrathecally injected with pcDNA (*n* = 6) or pcDNA‐TCTN2 (*n* = 6) vector. (A) BBB scoring was used to estimate the neurological function at 1, 6, 12, 24, and 48 h after SCI induction. (B) Forty‐eight hours later, the spinal tissue of mice was taken and the expression of TCTN2 and miR‐216b in spinal tissue of rats was examined by qRT‐PCR. (C) The P62, LC3I, and LC3II protein level in spinal tissue was analyzed with western blot 48 h after SCI. *P < 0.05 compared with pcDNA. The error bars indicate SD. The experiments were repeated three times. Comparisons between the two groups were analyzed with Student's *t* test.

The article "Overexpression of lncRNA TCTN2 protects neurons from apoptosis by enhancing cell autophagy in spinal cord injury" was published in 2019. Journal: FEBS Open Bio.

## Discussion

SCI is a serious neurological trauma, but its pathogenesis and the key influencing factors have not been precisely illuminated 18. Neuronal apoptosis is a main factor in neuronal loss and is widely considered to be implicated in the development of SCI 19. In addition, neuronal autophagy has also been shown to decrease neuronal damage and promote locomotor restoration by restraining of apoptosis after SCI in rats 8, 20. In the current study, we utilized an *in vivo* SCI model and human neurons to clarify the role of autophagy in SCI and its interrelationship with apoptosis, in which the function of lncRNA TCTN2 is initially highlighted. It can be summarized that TCTN2 increases autophagy by targeting the miR‐216b–Beclin‐1 pathway to control neuronal apoptosis, thus relieving spinal cord injury. Our study may provide new promising targets for SCI treatment and prognostic evaluation.

A regulatory effect of lncRNAs on cell autophagy or apoptosis has been validated in human disease. For instance, lncRNA MALAT1 promotes autophagy resulting in suppression of tumor cell apoptosis in multiple myeloma 21. LncRNAs also have been reported to regulate SCI initiation and progression, mostly by affecting cell autophagy or apoptosis. LncRNA SCIR1 down‐regulation has been proven to play a detrimental role in the pathophysiology of traumatic SCI through stimulating astrocyte proliferation and migration 22. In acute SCI, knockdown of lncRNA BDNF‐AS suppresses neuronal cell apoptosis 23, while lncRNA XIST contributes to neuronal apoptosis in rat SCI 17. Suppression of lncRNA Sox2ot decreases apoptosis and autophagy to inhibit H_2_O_2_‐induced PC‐12 cell injury and injury in spinal cord 24. The present study illustrates that lncRNA TCTN2 represses neuronal apoptosis by increasing autophagy, revealing a neuroprotective role of TCTN2 in SCI to benefit locomotor recovery of SCI rats. This result is in line with the significance of the TCTN2 gene in neural tube development 14.

Most lncRNAs show regulatory effects in disease initiation and progression by serving as the competing endogenous RNAs of miRNAs 25. By competitively binding miR‐494, lncRNA XIST contributes to neuronal apoptosis in rat SCI, participating in the pathogenesis of SCI 17. MALAT1 exhibits a neuroprotective role in spinal cord ischemia–reperfusion injury through miR‐204 regulation 26. The present study innovatively identifies miR‐216b as a down‐stream target of lncRNA TCTN2, uncovering the critical relationship between TCTN2 and miR‐216b in human disease. MiR‐216b is a member of the miRNAs that negatively regulates gene expression to take part in human diseases such as nasopharyngeal carcinoma 27, cervical cancer 28, and hepatocellular carcinoma 29, acting as a tumor suppressor. Moreover, miR‐216b has been noted to modulate autophagy and reduce LC3II in hepatocellular carcinoma cells, and miR‐216b represses autophagy and apoptosis through Beclin‐1 in human Tenon's capsule fibroblasts induced by hydroxycamptothecin 12, 30. Beclin‐1 is a key autophagy‐related protein and apoptosis regulator 31, and Beclin‐1‐mediated autophagy has been reported to protect spinal cord neurons from apoptosis 10, demonstrating its neuroprotective role in SCI. Our study confirms once more the function of Beclin‐1 in autophagy, apoptosis, and SCI progression, but the role of miR‐216b in affecting neuronal apoptosis and SCI, achieved by controlling Beclin‐1, was discovered for the first time.

The article "Overexpression of lncRNA TCTN2 protects neurons from apoptosis by enhancing cell autophagy in spinal cord injury" was published in 2019. Journal: FEBS Open Bio.

In summary, these findings highlight the regulatory effects of lncRNA TCTN2 on neuronal autophagy and apoptosis by targeting the miR‐216b–Beclin‐1 pathway, which is beneficial for SCI improvement, offering novel insights for SCI amelioration and neurological function recovery after SCI. However, some limitations still exist in this work. In the first place, more potential targets of lncRNA TCTN2 need to be explored to seek the optimal miRNA that has the maximal influence on neuronal autophagy, apoptosis, and SCI. In addition, many other targeting genes of miR‐216b and the other competing endogenous RNAs of miR‐216 also deserve further investigation in the future.

## Conflict of interest

The authors declare no conflict of interest.

## Author contributions

CW conceived and designed this study, and contributed to the acquisition of the data and the preparation of the manuscript. XR designed the study, analyzed the data, drafted and made crucial revision of the manuscript for important intellectual content. YN contributed to the conception of the study, collection and analysis of the data, manuscript editing and revision. All the authors approved the final version.
